# Effects of Stone Removal via Different Approaches in the Treatment of Incarcerated Upper Ureteral Calculi: A Comparative Study

**DOI:** 10.1155/2022/7651215

**Published:** 2022-07-08

**Authors:** Xiaoliang Yuan, Hanping Wei, Xiaowu Liu, Zhimin Jiao, Tingchun Wu, Honglei Shi

**Affiliations:** Department of Urology, Changzhou Wujin Peoples Hospital, Changzhou, Jiangsu 213000, China

## Abstract

**Objective:**

The aim of this study is to investigate the clinical effects of percutaneous nephrolithotomy and transurethral ureteroscopic lithotripsy in the treatment of incarcerated upper ureteral calculi.

**Methods:**

This study retrospectively reviewed 400 patients with incarcerated upper ureteral calculi admitted to the hospital from January 2016 to December 2021. Among them, 200 patients treated with percutaneous nephrolithotomy were included in the percutaneous group and 200 patients treated with transurethral ureteroscopic lithotripsy were included in the transurethral group. Perioperative indicators and stone clearance rates on day 7 and 1 month after operation and the reoperation rate were compared between the two groups. The incidence of postoperative complications was recorded.

**Results:**

The operation time and postoperative hospital stay of the percutaneous group were longer than those of the transurethral group (*P* < 0.05). There was no significant difference in intraoperative blood loss, 24 h postoperative pain score, stone clearance rates on day 3 and day 14 after operation, or the reoperation rate between the two groups (*P* > 0.05). Postoperative complications in the two groups were mainly grade I and II. The total incidence of complications in the percutaneous group was significantly lower than that in the transurethral group (*P* < 0.05).

**Conclusion:**

Both percutaneous nephrolithotomy and transurethral ureteroscopic lithotripsy are effective in the treatment of incarcerated upper ureteral calculi. The former can reduce the incidence of postoperative complications, but the operation time and postoperative hospital stay are longer.

## 1. Introduction 

Incarcerated upper ureteral calculi are one of the common clinical diseases of the urinary system, with lumbar colic, hematuria, and fever as the main clinical symptoms. In the past, conservative treatment, extracorporeal shock wave lithotripsy, and open surgery were used to treat incarcerated upper ureteral calculi, but the clinical effect was limited [1]. With the development of endoscopic technology, various endoscopic minimally invasive procedures have become the main methods for the treatment of incarcerated upper ureteral calculi, including percutaneous nephrolithotomy, transurethral ureteroscopic lithotripsy, etc. [2,3]. However, the clinical efficacy of the abovementioned two commonly used surgical methods has been controversial and no consensus has been attained [4]. In order to further clarify the clinical effect of percutaneous renal ureteral lithotripsy and transurethral ureteral lithotripsy in the treatment of incarcerated upper ureteral calculi, this study retrospectively analyzed the clinical data of 400 patients with incarcerated upper ureteral calculi, the operative indicators, stone clearance rate, complications, etc., and can provide reference for the selection of surgical methods for the clinical treatment of incarcerated upper ureteral calculi.

## 2. Materials and Methods

### 2.1. General Information

The clinical data of 400 patients with incarcerated upper ureteral calculi who were treated in our hospital from January 2016 to December 2021 were retrospectively analyzed. The inclusion criteria were as follows: ① Ultrasound or CT confirmed that the stone was located in the upper ureter of one side; ② the stone obstruction time was more than 2 months, which was in line with the indication for surgery; and ③ the patient was not limited by gender, and the age was more than 18 years old. The exclusion criteria were as follows: ① patients with kidney stones requiring primary surgical treatment; ② patients with middle and lower ureteral calculi; ③ patients with severe urethra or ureteral stricture; ④ patients with severe urinary tract infection; and ⑤ patients with major organ dysfunction. Among them, 200 patients were treated with percutaneous renal ureteral lithotripsy (percutaneous renal group) and 200 patients were treated with transurethral lithotripsy (transurethral group). This study was approved by the hospital ethics committee, and there was no statistical significance in the general clinical data between the two groups (*P* > 0.05) as shown in Table 1.

### 2.2. Treatment Methods

Percutaneous kidney group: The patients received percutaneous nephrolithotomy. The patient was placed in the lithotomy position, and after anesthesia was routinely sterilized and draped, the affected ureter was examined by a transurethral ureteroscope, and the F6 ureteral catheter was placed along the guide wire into the affected ureter. The catheter was retained and the catheter was properly fixed. The body position was changed to the prone position, the puncture point (the posterior axillary line to the subscapular line, the 10th intercostal space to the 12th rib) was determined, and the puncture needle was inserted at the puncture point under the guidance of ultrasound wire and the puncture needle withdrawn. The fascia dilator was used for step-by-step expansion along the guide wire (F8∼F18). When the channel was expanded to F18, the working sheath was indwelled, and the ureteroscope was inserted through the percutaneous renal microchannel for laser lithotripsy and lithotripsy. After the microscopic examination showed no residual stones, the double J tube was indwelled, the ureteroscope was withdrawn, the urinary catheter was set, and the operation was completed.

Transurethral group: The patients received transurethral lithotripsy. The patient was placed in the lithotomy position, and after anesthesia was routinely disinfected and draped, the transurethral ureteroscope was directly placed into the bladder, and the zebra guide wire was inserted into the ureter on the affected side through the urethra and the ureteroscope was placed along the guide wire into the upper ureteral calculus position, with a 200 *μ*m implant. Through optical fiber and laser lithotripsy, after the stones were cleaned, a 5F ureteral stent was indwelled, the ureteroscope was withdrawn, the urinary catheter was set, and the operation was completed.

### 2.3. Observation Indicators

The observation indicators are as follows: ①Perioperative indicators: The perioperative indicators such as operation time, intraoperative blood loss, postoperative 24-hour pain score, and postoperative hospitalization time were compared between the two groups. The higher the score, the more pain the patient feels. ② Stone removal status: The stone removal rate and secondary operation rate (referring to nonconcurrent invasive operations) were compared between the two groups at 7d and 1 month after operation. ③ The postoperative complications of the patients were recorded, including pain, fever, nausea and vomiting, urinary tract infection, ureteral stricture, etc., within a month, and the complications were graded with reference to the modified Clavein grading standard [5].

### 2.4. Statistical Processing

SPSS 20.0 statistical software was used to analyze the data. The measurement data is expressed as independent sample t-test, which is used for the comparison between the two groups the enumeration data were expressed as *n* (%), and carry out the *χ*2 test. *P* < 0.05 was considered statistically significant.

## 3. Results

### 3.1. Comparison of Perioperative Indicators between the Two Groups of Patients

The operation time and postoperative hospital stay in the percutaneous renal group were longer than those in the transurethral group (*P* < 0.05). There was no significant difference in intraoperative blood loss and 24 h postoperative pain score between the two groups (*P* > 0.05) as shown in Table 2.

### 3.2. Comparison of Stone Clearance between the Two Groups of Patients

There was no significant difference in the stone clearance rate and secondary operation rate at 7 d and 1 month after operation between the two groups (*P* > 0.05) as shown in Table 3.

### 3.3. Comparison of Postoperative Complications between the Two Groups of Patients

No serious complications (Grade III, IV, V) occurred in all patients. Grade I complications were mainly pain, fever, and vomiting. Grade II complications were mainly urinary tract infection and ureteral stricture. The total incidence of complications in the percutaneous group was significantly lower than that in the transurethral group, and the difference was statistically significant (*P* < 0.05) as shown in Table 4.

## 4. Discussions

Kidney stones descending and draining into the ureter are the main reasons for the formation of ureteral stones. When the stones are larger in diameter and irregular in shape, they are easily incarcerated in the upper ureter, forming incarcerated upper ureter stones. It can cause ureteral obstruction, urinary tract infection, hydronephrosis, etc., and eventually lead to the loss of renal function [6]. Therefore, ureteral calculi should be removed in time, the obstruction should be relieved, and the renal function of the affected side should be protected.

Surgical treatment is an important method for clinical treatment of incarcerated upper ureteral calculi. Among the commonly used percutaneous ureteroscopic lithotripsy and transurethral calculi, percutaneous renal ureteral calculi in the treatment of intrarenal and upper ureteral calculi have a clear curative effect, but the ureter is tortuous or narrow, which makes the operation difficult. The requirements are higher [7]. However, transurethral lithotripsy is simple to operate but has a high postoperative complication rate and poor efficacy [8]. The efficacy of the two methods in the treatment of incarcerated upper ureteral calculi has been controversial. This study compared the clinical effects of two surgical methods for the treatment of incarcerated upper ureteral calculi. The results of the study showed that the operation time and postoperative hospital stay in the percutaneous renal group were longer than those in the transurethral group, but the intraoperative blood loss and postoperative 24-hour pain were significantly higher. There was no significant difference in the score comparison, suggesting that percutaneous renal ureteral lithotripsy has no obvious advantages in terms of operation time and postoperative hospital stay. Li Lin et al [9] compared the efficacy of minimally invasive percutaneous nephrolithotomy and ureteroscopic lithotripsy in the treatment of upper ureteral incarcerated calculi and found that percutaneous nephrolithotomy may prolong the operation time and the patient's hospital stay. It is believed that the particularity of the location of incarcerated upper ureteral stones and the difference in stone morphology will increase the difficulty of operation and prolong the operation time, and the indwelling operation of nephrostomy tube after operation will further prolong the operation time and hospitalization time of patients. Comparing the stone removal conditions of the two groups of patients, it can be seen that there was no significant difference in the stone removal rate and the second operation rate between the two groups at day 7 and 1 month after operation, which is consistent with the results of the previous study [10]. It has a good effect in the treatment of incarcerated upper ureteral calculi. The diameter of the distal end of the ureter is smaller than that of the proximal end. When percutaneous nephroureteroscopy is used for lithotripsy, the probability of intraoperative calculus movement is low, and the lithotripsy effect is guaranteed. However, some scholars' studies [11] found that the effect of transurethral lithotripsy therapy was significantly better than that of percutaneous renal ureteral lithotripsy, which was considered to be related to different stone loads, stone locations, and operator's operation levels in different patients. This study found that the postoperative complications of the two groups were mainly Grade I and II and the total incidence of complications in the percutaneous renal group was significantly lower than that in the transurethral group, suggesting that percutaneous renal ureteral lithotripsy can reduce postoperative complications in patients' incidence. In transurethral lithotripsy surgery, in order to maintain a clear vision, it is often necessary to inject water into the working channel, so that the perfusion pressure in the channel is high, and continuous long-term high-pressure perfusion will increase the risk of postoperative bacterial infection and bacteremia. The postoperative fever rate increased [12]. After lithotripsy, powdered stones need to be slowly excreted by indwelling ureteral stents, and the cycle is long, which also increases the risk of infection to a certain extent. In addition, when the ureteroscope moves in the cavity, patients with poor ureteral conditions are more susceptible to mechanical damage and ureteral stenosis is induced under the action of inflammation and tissue fibrosis. The study by Lv Wanghua et al. [13] also found that compared with ureteroscopic lithotripsy, patients who received percutaneous nephrolithotomy had a lower incidence of complications and believed that percutaneous nephrolithotomy was safer, which is beneficial to the prognosis of patients.

In conclusion, percutaneous renal ureteral lithotripsy and transurethral ureteral lithotripsy have good effects in the treatment of incarcerated upper ureteral calculi. Percutaneous renal ureteral stone removal can reduce the incidence of postoperative complications, but the operation time and postoperative hospital stay are longer.

## Figures and Tables

**Table 1:** Comparison of general clinical data of two groups of patients (n (%)).

Indexes	Number of cases	Percutaneous kidney group (*n* = 200)	Transurethral group (*n* = 200)	*χ* ^*2*^ */t*	*P*
Gender	Male	123 (61.50)	119 (59.50)	0.167	0.682
	Female	77 (38.50)	81 (40.50)		
Age (years)		53.34 ± 10.35	53.00 ± 9.91	0.341	0.734
The diameter of the stone (mm)		10.18 ± 2.09	10.28 ± 3.12	0.377	0.707
Stone location	Left side	105 (52.50)	113 (56.50)	0.645	0.422
	Right side	95 (47.50)	87 (43.50)		
Stone CT value (HU)		771.14 ± 215.16	786.24 ± 201.91	0.724	0.470

**Table 2:** Comparison of perioperative indicators between the two groups of patients (n, $\overset{-}{x}\pm s$)

Group	Operation time (min)	Intraoperative blood loss (ml)	24-h Postoperative pain score (score)	Postoperative hospital stay (d)
Percutaneous kidney group (*n* = 200)	42.37 ± 9.88	18.64 ± 5.98	5.12 ± 1.22	5.93 ± 1.96
Transurethral group (*n* = 200)	31.86 ± 10.59	17.95 ± 4.55	4.89 ± 1.42	3.68 ± 1.06
*T*	10.259	1.299	1.697	14.282
*P*	<0.001	0.195	0.091	<0.001

**Table 3:** Comparison of stone clearance between two groups of patients (*n*, %).

Group	Stone clearance rate at 7 d postoperatively	Stone clearance rate at 1 month postoperatively	Secondary surgery rate
Percutaneous kidney group (*n* = 200)	179 (89.50)	197 (98.50)	3 (1.50)
Transurethral group (*n* = 200)	181 (90.50)	195 (97.50)	4 (2.00)
*χ* ^*2*^	0.111	0.510	0.145
*P*	0.739	0.475	0.703

^*∗*^ row Fisher's exact probability test.

**Table 4:** Comparison of postoperative complications between the two groups of patients (n,%).

Group	Grade I			Grade II		Overall incidence
	Pain	Fever	Vomiting	Urinary tract infection	Ureteral stricture	
Percutaneous kidney group (*n* = 200)	8 (4.00)	5 (2.50)	3 (1.50)	2 (1.00)	1 (0.50)	19 (9.50)
Transurethral group (*n* = 200)	10 (5.00)	9 (4.50)	5 (2.50)	5 (2.50)	4 (2.00)	33 (16.50)
*χ* ^*2*^						4.332
*P*						0.037

## Data Availability

The data used and/or analyzed during the current study are available from the corresponding author upon request.
